# A Deep Learning Approach for Mild Depression Recognition Based on Functional Connectivity Using Electroencephalography

**DOI:** 10.3389/fnins.2020.00192

**Published:** 2020-04-01

**Authors:** Xiaowei Li, Rong La, Ying Wang, Bin Hu, Xuemin Zhang

**Affiliations:** ^1^Gansu Provincial Key Laboratory of Wearable Computing, School of Information Science and Engineering, Lanzhou University, Lanzhou, China; ^2^CAS Center for Excellence in Brain Science and Intelligence Technology, Shanghai Institutes for Biological Sciences, Chinese Academy of Sciences, Shanghai, China; ^3^Beijing Institute for Brain Disorders, Capital Medical University, Beijing, China; ^4^Beijing Key Laboratory of Applied Experimental Psychology, National Demonstration Center for Experimental Psychology Education, Faculty of Psychology, Beijing Normal University, Beijing, China; ^5^State Key Laboratory of Cognitive Neuroscience and Learning and IDG/McGovern Institute for Brain Research, Beijing Normal University, Beijing, China; ^6^Center for Collaboration and Innovation in Brain and Learning Sciences, Beijing Normal University, Beijing, China

**Keywords:** EEG, functional connectivity, convolutional neural network, mild depression, classification

## Abstract

Early detection remains a significant challenge for the treatment of depression. In our work, we proposed a novel approach to mild depression recognition using electroencephalography (EEG). First, we explored abnormal organization in the functional connectivity network of mild depression using graph theory. Second, we proposed a novel classification model for recognizing mild depression. Considering the powerful ability of CNN to process two-dimensional data, we applied CNN separately to the two-dimensional data form of the functional connectivity matrices from five EEG bands (delta, theta, alpha, beta, and gamma). In addition, inspired by recent breakthroughs in the ability of deep recurrent CNNs to classify mental load, we merged the functional connectivity matrices from the three EEG bands that performed the best into a three-channel image to classify mild depression-related and normal EEG signals using the CNN. The results of the graph theory analysis showed that the brain functional network of the mild depression group had a larger characteristic path length and a lower clustering coefficient than the healthy control group, showing deviation from the small-world network. The proposed classification model obtained a classification accuracy of 80.74% for recognizing mild depression. The current study suggests that the combination of a CNN and functional connectivity matrix may provide a promising objective approach for diagnosing mild depression. Deep learning approaches such as this might have the potential to inform clinical practice and aid in research on psychiatric disorders.

## Introduction

Depression is a global public health problem, which has a relatively high lifetime prevalence, ranging from 2 to 15%, and is associated with significant morbidity (Ustun and Chatterji, 2001; Üstün et al., 2004). According to the latest data from the World Health Organization (2017)^1^, more than 300 million people are now living with depression^1^. Presently, the most widely used methods for depression diagnosis are based on Beck’s Depression Inventory (BDI), the patient’s self-report, the doctor’s clinical experience, or some combination thereof. However, the accuracy of this diagnosis is often influenced by the doctor’s proficiency and patient’s cooperation, both of which are highly subjective. Critically, a subset of depression–mild depression–receives far less attention than does depression, despite being more common than depression and often increasing in severity over time (Volz and Laux, 2000). This lack of attention leads to missed early detection and treatment and increases the mortality risk and likelihood that mild depression will evolve into major depression (Fogel et al., 2006; Lyness et al., 2006). Additionally, mild depression is not only a mental illness but also often a social problem (Li et al., 2016b). Therefore, studies of methods that might improve the early detection and treatment of mild depression are both necessary and meaningful.

With the emergence of more and more studies of depression using functional brain imaging, it is becoming clear that this psychopathology might be relevant to the distributed properties of large-scale cortical systems across many functionally connected cortical regions (Spence, 1995; Dalgleish, 2004; Wang et al., 2012). Recent studies have provided further evidence that depressed individuals tend to have altered brain functional connectivity, such as significantly decreased functional connectivity between right posterior insula and a series of sensory cortices (Hu et al., 2019), decreased brain activity in the dorsolateral prefrontal cortex, superior temporal gyrus, posterior precuneus, and posterior cingulate (Zhong et al., 2016), and increased subgenual cingulate–thalamic connectivity (Ajilore et al., 2015). To examine the functional connectivity of the brain, various metrics have been used, including coherence, correlation, phase locking value, and phase lag index, among others.

Electroencephalography (EEG) coherence is an effective measure of functional cortical connectivity and is used to calculate linearly dependent interactions between the frequencies of EEG signals derived from two electrodes or brain regions (Andrew and Pfurtscheller, 1996; Pfurtscheller and Andrew, 1999). This measure results in a symmetrical, two-dimensional (2D) matrix. High coherence between two EEG signals reflects synchronized neuronal oscillations (suggesting functional integration between neural populations), while low coherence indicates independently active populations (suggesting functional segregation) (Murias et al., 2007). Using EEG coherence to study the brain activity of patients with depression (Li et al., 2017), as well as those with Alzheimer’s disease (AD) (Wada et al., 1998) and Parkinson’s disease (Teramoto et al., 2016), has been quite successful. For example, Murias et al. (2007) observed an elevated EEG theta coherence in the frontal and temporal regions of the left hemisphere in individuals with autism spectrum disorder. In a study that used EEG coherence to assess resting state functional connectivity, Teramoto et al. (2016) found a decreased resting state functional connectivity between the frontal and parietal cortices, especially in the left hemisphere, of patients with Parkinson’s disease. Yingjie et al. (Li et al., 2015) further used EEG coherence to investigate differences in brain functional networks between patients with depression and healthy controls, while they were processing emotional stimuli. The authors found that global EEG coherence in the gamma band was significantly higher in patients with depression than it was in healthy controls.

Correlation is an alternative method of calculating functional connectivity matrices and is often used to estimate the level of linear dependence between two electrode channels. In a study by Zhang et al. (2018) that measured functional connectivity, the authors calculated the Pearson correlation coefficients of the power spectral densities for the delta, theta, alpha, beta, and gamma bands. Following this, they constructed a square correlation matrix for each participant and each frequency band. Finally, the functional brain networks of healthy controls and patients with major depressive disorder (MDD) were constructed using the correlation matrix. The results revealed that compared to healthy controls, the patients with MDD showed significant randomization of the global network metrics.

A statistical method known as “phase synchronization” can also be used to measure coordinated activation across different brain regions. In biological signals, such as EEG time series, synchronization is measured by calculating the phase locking value (PLV). Mormann et al. (2000) reported on the application of phase synchronization methods to biological time series data representative of brain electrical activity in patients with epilepsy. They observed characteristic spatial and temporal shifts in synchronization that appeared to be strongly related to pathological activity. In particular, the authors reported distinct differences in the degree of synchronization between recordings from seizure-free intervals and those from the intervals just before an impending seizure.

The phase lag index (PLI) is another measure of asymmetry in the distribution of phase differences between two signals. The PLI is an alternative measure of statistical interdependencies between time series that reflects the strength of their coupling by detecting consistent, non-zero phase lag between the two times series. Stam et al. (2007) found that PLI performed well for detecting relative increases in synchronization between the pre-seizure and seizure epochs. In addition, upon analyzing the EEG signals, the authors found that the average PLI in the beta band was significantly lower in patients with AD (15 subjects) than it was in healthy controls (15 subjects).

The current mainstream method for studying brain functional connectivity is to convert a functional connectivity matrix into a graph via graph theory analysis. After completing a characterization of the topological properties of the graph, the clustering coefficient and characteristic path length–two indices that characterize a graph and correspond to the two basic principles of brain functional organization, namely, functional separation and integration (Friston, 2009), respectively–are used to distinguish between patients with neurological disorders and healthy controls. In addition, these two indices can comprehensively reflect the small-world characteristics of the network. Randomization of network topology and distribution of the small-world network architecture have been consistently shown in AD, schizophrenia, and depression. Stam et al. (2006) found that the characteristic path length in AD patients was significantly longer than that in healthy controls and demonstrated that AD is characterized by loss of small-world network characteristics. Rubinov et al. (2009) found a randomization of the small-world network structure in schizophrenia. One EEG study showed that the loss of small world characteristics in the sleep functional brain network in MDD indicates a disruption of topological organization caused by this disease (Zhang et al., 2011). In addition, Leistedt et al. (2009) reported that the healthy controls’ neural network is closer to the ordered part of the rewiring scale, while the depressed patients’ brain network during sleep is closer to the random part of the scale. Although changes in brain function connectivity in MDD have been known, the functional brain network structure of mild depression is unclear. Therefore, we analyzed the functional brain network of mild depression through graph theory.

Deep neural networks have recently achieved great success in the widespread application of large-scale image- (Hinton et al., 2012), video- (Karpathy et al., 2014), and text-based recognition tasks (Hermann et al., 2015; Zhang and Lecun, 2015). Convolutional neural networks (CNNs) lie at the core of the best current architecture processing methods for both image and video data, primarily due to the advantages of CNNs in processing 2D input data (Cecotti and Graser, 2011). CNN has good performance in the field of biological image classification, and the features learned from CNN are often better than handcrafted features (Bello-Cerezo et al., 2019). The studies of Nanni et al. (2019a; 2019b) show that ensemble system of handcrafted and learned features can boost the performance of CNN in bioimage classification. In neural signal classification, several studies have used different methods to convert EEG signals into image representations. One, in particular, used the short-term Fourier transformation method to convert EEG time series into 2D images and combined 1D CNNs and stacked autoencoders to classify EEG motor imagery signals (Tabar and Halici, 2016). This approach yielded a 9% improvement over the winning algorithm. A new representation of EEG signals was proposed by Bashivan et al. (2015) that preserves the structure of EEG data across space, time, and frequency bands. In this approach, 3D electrode locations were projected onto a 2D surface using azimuthal equidistant projection, and the spectral power within three prominent frequency bands was extracted for each location. This was then used to form topographical maps that were subsequently combined to form three-channel images. Finally, these three-channel images were input into a deep convolutional recurrent neural network to further classify the EEG signals. Inspired by these studies and the powerful ability of CNNs to process 2D data, we innovatively applied a CNN to the 2D data form of functional connectivity matrices and constructed a classification model for mild depression as a depression recognition method other than graph theory.

In addition, research on facial emotion processing plays a significant role in the study of emotion and cognition in patients with depression. For example, David et al. (Rubinow and Post, 1992) conducted an experiment where 17 patients with depression and 31 healthy controls were asked to recognize seven affective states within images of facial expressions. The results revealed that patients with depression were significantly impaired in their ability to recognize facial affect; specifically, they made significantly (or nearly significantly) fewer correct matches for sad, happy, and interested face items. Similarly, James et al. (Cavanagh and Geisler, 2006) examined mood-relevant emotion processing in individuals with depression using event-related potentials. Mixed-model analyses of variance revealed significantly reduced P3 amplitudes and P3 latencies for happy faces in participants with depression. The authors interpreted these findings as providing evidence for a diminished cognitive processing ability during emotion discrimination in individuals with depression. Collectively, these studies reveal differences in the brain activity of patients with depression and healthy individuals during common face-processing tasks. Therefore, in the current study, we used a facial expression paradigm to investigate differences in brain functional connectivity between individuals with mild depression and healthy controls.

In the present study, we first studied the differences in the brain functional network between the mildly depressed group and the normal control group using graph theory. We calculated the four functional connectivity matrices of coherence, correlation, PLV, and PLI and converted them into binary undirected graphs. We calculated the characteristic path length, clustering coefficient, and the small-world properties of the brain functional network of the two groups to investigate the differences in these indices between two groups. Then, we proposed a novel approach aimed at improving the ability to recognize individuals with mild depression. Inspired by the proven utility of CNNs in image processing, we used a CNN to process EEG signals. EEG time series signals were converted into images through calculating functional connectivity matrices, and then these images from the two groups were used to classify individuals with mild depression and healthy controls in a CNN.

## Materials and Methods

### Network Analysis

#### Coherence Analysis

Coherence is defined as the spectral cross-correlation between two signals normalized by their power spectrum. Coherence is computed mathematically as:

(1) $$C\,o\,h_{x\,y}\,\left(f\right)=\frac{\left|\frac{1}{n}\,\sum_{k=1}^{n}A\,x\,\left(f,k\right)\,A\,y\,\left(f,k\right)\,e^{i\,\left(\varphi_{x}\,\left(f,k\right)-\varphi_{y}\,\left(f,k\right)\right)}\right|}{\sqrt{\left(\frac{1}{n}\,\sum_{k=1}^{n}A_{x}^{2}\,\left(f,k\right)\right)\,\left(\frac{1}{n}\,\sum_{k=1}^{n}A_{y}^{2}\,\left(f,k\right)\right)}}$$

where *n* is the number of data points in a trial. *A* and *φ* are the amplitude and phase of the signal, respectively. The numerator term represents the cross-spectral density on a single trial between the signals *x* and *y* at frequency *f*. The denominator represents the square root of the product of the power estimates on a single trial of the signals *x* and *y* at frequency *f*.

The coherence can then be concisely defined as:

(2) $$C\,o\,h_{x\,y}\,\left(f\right)=\frac{\left|S\,x\,y\,\left(f\right)\right|}{\sqrt{S\,x\,x\,\left(f\right)\,S\,y\,y\,\left(f\right)}}$$

where Sxy(f) is the cross-spectral density of the signal, and *Sxx*(*f*) and *Syy*(*f*) are the power spectral density of signals *x* and *y*, respectively. Values of *Coh*_*xy*_will always satisfy 0 ≤ *Coh*_*xy*_(*f*) ≤ 1, where 0 represents no coupling, and 1 indicates maximum linear interdependence between two signals.

#### Correlation Analysis

Correlation (Pearson correlation coefficient) is used to estimate the level of linear dependence between two electrode channels in the time domain. The correlation is given by the following:

(3) $$C\,o\,r\,r_{x\,y}=\frac{C\,o\,v\,\left(x,y\right)}{\sigma_{x}\,\sigma_{y}}$$

where *Cov*(*x*,*y*) is the covariance between electrodes *x* and*y*, σ_*x*_and σ_*y*_ are the standard deviations of the electrodes *x* and *y*, respectively. *Corr*_*xy*_ has a value between 1 and −1, where 1 is a total positive linear correlation, 0 is no linear correlation, and −1 is a total negative linear correlation. The greater the absolute value of *Corr*_*xy*_, the stronger the correlation.

#### Phase Locking Value Analysis

The PLV (Mormann et al., 2000) assumes that the signal amplitude and phase are statistically independent, and thus, only the phase synchronization is used to estimate a possible functional interaction between the EEG signals of two channels. When Ax(.,.) = Ay(.,.) = 1 in Eq. (1), the PLV is obtained (Lachaux et al., 1999), as follows:

(4) $$\begin{array}{c} P\,L\,V_{x\,y}\,\left(f\right)=\frac{\left|\frac{1}{n}\,\sum_{k=1}^{n}1\,x\,\left(f,k\right)\,1\,y\,\left(f,k\right)\,e^{i\,\left(\varphi_{x}\,\left(f,k\right)-\varphi_{y}\,\left(f,k\right)\right)}\right|}{\sqrt{\left(\frac{1}{n}\,\sum_{k=1}^{n}1_{x}^{2}\,\left(f,k\right)\right)\,\left(\frac{1}{n}\,\sum_{k=1}^{n}1_{y}^{2}\,\left(f,k\right)\right)}}\\ =\left|\frac{1}{n}\,\sum_{k=1}^{n}e^{i\,\left(\varphi_{x}\,\left(f,k\right)-\varphi_{y}\,\left(f,k\right)\right)}\right| \end{array}$$

The value of PLV is between 0 and 1, where 0 represents a lack of synchronization, and 1 represents perfect phase synchronization.

#### Phase Lag Index Analysis

The PLI (Stam et al., 2007) is a measure of the asymmetry of the distribution of phase differences between two EEG signals and is defined as follows:

(5) $$P\,L\,I_{x\,y}\,\left(f\right)=\left|\frac{1}{n}\,\sum_{k=1}^{n}s\,i\,g\,n\,\left(\phi_{x}\,\left(f,k\right)-\phi_{y}\,\left(f,k\right)\right)\right|$$

where *n* is the number of data points, and ϕ_*x*_(*f*,*k*)−ϕ_*y*_(*f*,*k*) represents the phase synchronization between the signals in channels *x* and *y* at the frequency *f*. It is essential to know the instantaneous phase of the two signals involved, which can be achieved using the analytical signal based on the Hilbert transform (Bruns, 2004), to compute the phase synchronization. The *PLI*_*xy*_(*f*) ranges between 0 and 1, where 1 indicates perfect phase synchronization and 0 indicates either no coupling or coupling with a phase difference centered around 0 mod π. PLI, contrary to the other methods, basically disregards perfect coupling (zero phase) or phase opposition coupling, which cannot be distinguished from no coupling.

Four kinds of metrics, coherence, correlation, PLV, and PLI, were calculated using all 128 EEG channels through the Neurophysiological Biomarker Toolbox^2^. For each trial, four 128 × 128 matrices were obtained (128 was the number of EEG channels). For each kind of metric, we considered the following EEG bands: delta (1–4 Hz), theta (4–8 Hz), alpha (8–13 Hz), beta (13–30 Hz), and gamma (30–70 Hz).

#### Complex Network Analysis

Applying graph theoretical analysis to a functional connectivity matrix is to convert the matrix into a binary undirected graph. The functional connectivity matrix can be converted to a graph by considering a threshold T. If the functional connectivity metric between a pair of channels exceeds T, then there is an edge, otherwise there is no edge. The choice of T has an important impact on the constructed graph, i.e., a low *T*-value will result in a densely connected network, while a large *T*-value will result in a sparse network. Since there is no unique method to select the appropriate threshold, we studied the entire range of values of *T* (0 < *T* < 1, with increments of 0.025 for coherence, correlation, and PLV and 0.005 for PLI) and repeated the full analysis for each value of *T*.

Once we converted the functional connectivity matrix into a graph, the next step is to characterize the graph in terms of its characteristic path length L and its cluster coefficient C. These two indices correspond to the two basic principles of brain function organization, that is, functional integration and segregation (Friston, 2009). Functional integration reflects the brain’s ability to organize and combine information from different brain regions, and could be well measured by the characteristic path length L, which is obtained by calculating the average shortest path length between all pairs of nodes. Functional segregation reflects the ability to process information in a specialized way. Clustering coefficient C is often used to measure functional segregation. “C quantifies the number of connections between the nearest neighbours of a node as proportion of the maximum possible number of connections” (Strogatz, 2001). After clustering coefficients of all nodes are calculated, the average is taken as the clustering coefficient of the network.

To establish the network topology characteristics, the ratios C/Cr and L/Lr are calculated as a function of the threshold T, where Cr and Lr represent the values of C and L for matched random networks. Random networks have the same nodes and connectivity as the original network, whereas their choice of connected nodes is completely random. Following the previous studies (Watts and Strogatz, 1998; Stam et al., 2006; Li et al., 2015) that generated 20 random networks, 20 matched random networks are generated here for each actual network of each subject, and their average Cr and Lr are calculated to compare with the actual network. When values of C/Cr are significantly greater than 1, while the values of L/Lr are close to the value of 1, the small-world network organization is evident. In addition, Humphries et al. (2005) defined a single scalar index S to quantify the “small-world-ness” of a network, $S=\frac{\gamma }{\lambda }=\frac{C/C_{r}}{L/L_{r}}$, and a value of S greater than 1 is often used as a simple indicator of small-world organization.

The software used in this study was the Brain Connectivity Toolbox (Rubinov and Sporns, 2010) for calculating two graph theoretical measurements.

### Convolutional Neural Network

#### Input

We used only the upper triangular part of the 128 × 128 functional connectivity matrices due to the symmetry of matrices and computational efficiency of neural networks. This triangular part contains 8,256 elements, of which 128 are on the diagonal. As the elements on the diagonal are the coherence/correlation/PLV/PLI values between an electrode and itself, we excluded these 128 elements. Since the input to the CNN is generally square, we organized the remaining 8,128 elements into a square and made the size of the square as small as possible. In addition, considering that the functional connectivity metric located in the last part of the upper triangle is calculated based on the electrodes distributed on the face, they are more affected by myoelectricity and ocular electricity. We, thus, organized the 8,128 elements line by line into a 90 × 90 matrix and discarded the last 28 elements, which are calculated based on the eight electrodes E121, E122, E123, E124, E125, E126, E127, E128. The transformation process is depicted in Figure 1. A new 90 × 90 matrix was transformed into a single-channel image and served as the CNN’s input. It is worth mentioning that the elements in the functional connectivity matrix are arranged according to the increasing electrode number, and the neighborhood relationship between the electrodes did not represent the neighborhood information of 128 electrodes on HydroCel Geodesic Sensor Net. In other words, the location information of the electrodes was not preserved in the functional connectivity matrix. In addition, studies such as those mentioned in this review (De Aguiar Neto and Rosa, 2019) involve little information on the location of the electrodes when performing depression recognition. Similarly, in our study, the key piece of information for depression recognition is the functional connectivity value between the electrode pairs rather than the location of these values. So the element rearrangement during this transformation process will not have any obvious influence on mild depression recognition.

**FIGURE 1:** The transformation process of functional connectivity matrices. The first row represents the original functional connectivity matrices corresponding to 128 electrodes. The second row represents the new 90 × 90 matrices obtained by rearranging the elements in the upper triangle of the original functional connectivity matrices. From left to right are, the functional connectivity matrices for coherence, correlation, phase locking value, and the phase lag index.

In addition, inspired by the work of Bashivan et al. (2015), we merged the 90 × 90 single-channel functional connectivity matrices into an image with three channels. We used the three bands with the best classification performance for each functional connectivity matrix as the red, green, and blue channels to generate a three-channel image that was then fed into the CNN (Figure 2).

**FIGURE 2:** Three-channel input of the convolutional neural network (CNN). The three bands with the best classification performance among the five bands (delta, theta, alpha, beta, and gamma) of each type of functional connectivity matrix were used as the red (R), green (G), and blue (B) channels of the image to generate a three-channel image that was then used as input for the CNN.

#### Architecture

It is known that CNNs are multi-layer neural networks with several convolution–pooling layer pairs and a fully connected output layer (Tabar and Halici, 2016). A standard CNN (LeCun et al., 1990) is designed to recognize the shape in the images. As shown in Figure 3, the CNN model used here mainly included the following types of layers: convolution, pooling, activation function, fully connected layer, and softmax layer. Below, we provide brief descriptions of each of these.

**FIGURE 3:** Schematic structure of the convolutional neural network we constructed.

In simulating orientation-selective simple cells in the primary visual cortex of the brain (LeCun et al., 2010), convolution is considered to be an indispensable component of CNN frameworks. The input data *x* is a tensor with *K* channels. There are K′ filters of weights *W* generating *K*′output *y*, as shown in Eq. (6). In our network architecture, *K* = 1 or *K* = 3, *K*′ = 32.

(6) $$y_{i^{\prime }\,j^{\prime }\,k^{\prime }}=\sum_{i\,j\,k}w_{i\,j\,k\,k^{\prime }}\,x_{i+i^{\prime },j+j^{\prime },k}$$

In the present study, we adopted two stacked convolutional layers as the basic structure of the CNN. Each convolutional layer used 32 3 × 3 small filters with a convolution stride of one. Convolution layer inputs were padded with one pixel to preserve the spatial resolution after convolution.

Pooling was also an important operation in the CNN framework. Multiple pooling methods serve to simulate complex cells in the brain’s visual cortex (LeCun et al., 2010). In practice, the pooling method known as max pooling has been shown to work better than does average pooling. Specifically, max pooling calculates the max response of each feature map in a patch of size *p*×*p* as follows:

(7) $$y_{i\,j\,k}=\max\left\{y_{i^{\prime }\,j^{\prime }\,k}:i\leq i^{\prime }<i+p,j\leq j^{\prime }<j+p\right\}$$

Max pooling is performed over a 2 × 2-pixel window here with a stride of two.

Additionally, we selected a rectified linear unit as an activation function for our CNN model, since it has performed both accurately and quickly in other CNN models (Dahl et al., 2013; Donahue et al., 2014). Its output is given by the following formula:

(8) $$y_{i\,j\,k}=\max\left(0,x_{i\,j\,k}\right)$$

The max pooling layer is followed by a fully connected layer with 512 hidden cells, the last layer of which is a two-way softmax layer. The softmax layer is usually used for classification in CNN, and several classifications use several ways of softmax. In our study, since our goal is to distinguish between depression and normal subjects, that is, two classifications, we used two-way softmax. Softmax changes the output of the original neural network into a probability output to represent the probability that a sample belongs to different categories. Assuming that the output of the original neural network is *y*_1_,*y*_2_,…*y*_*n*_, then the output after softmax processing is:

(9) $$s\,o\,f\,t\,m\,a\,x\,{\left(y\right)}_{i}=\frac{e^{y_{i}}}{\sum_{j=1}^{n}e^{y_{j}}}$$

#### Training

Most of the code used in the present study was written in Python (version 3.5). The CNN model was trained and tested based on a lightweight library named Lasagne^3^, which was used for building and training the neural networks in Theano (Al-Rfou et al., 2016).

The network was trained with the Adam algorithm (Kingma and Ba, 2014), which has demonstrated a competitively fast convergence rate in the training of neural network (Bashivan et al., 2015). The learning rate was 10^–3^, and the decay rates of the first and second moments were 0.9 and 0.999, respectively. The weight initialization method we used was Xavier (Glorot and Bengio, 2010), which has been shown to be effective in network training (Jiao et al., 2018). We also used early stopping to monitor the performance of the model over the validation sets. Dropout (Hinton et al., 2012) with a probability of 0.5 was used across all fully connected layers. The effectiveness of this dropout to reduce overfitting in deep neural networks with millions of parameters has been shown previously (Krizhevsky et al., 2012) and in neuroimaging applications specifically (Plis et al., 2014). Because of implicit regularization imposed by smaller convolution filter sizes, the network requires fewer epochs to converge. Given this, our model was trained over 15 epochs with a batch size of 30.

## Experiments

### Participants

Fifty-one students (36 males, 15 females) aged between 18 and 24 were recruited from Lanzhou University and participated in the study. All of them had no prior history of psychopathology and had normal or corrected-to-normal vision. All participants were interviewed by psychologists after completing an investigation in the psychological screening system of Lanzhou University. According to psychologists, 24 of them were considered depressed, and the remaining 27 were healthy. Also, participants were asked to finish the Beck Depression Inventory test-II (BDI-II) (Beck et al., 1996) before experiment. Analysis of BDI-II showed that the BDI-II scores in the depression group ranges from 14 to 28, corresponding to mild depression, whereas the BDI-II scores of the healthy group were all lower than 13. In order to ensure that the number of samples was balanced for the two groups, 24 healthy participants were selected to comprise our control group. Table 1 shows the demographic characteristics and BDI-II scores of the two groups. This study was approved by the Ethics Committee of Lanzhou University Second Hospital (reference number: 2015A-037) and was conducted in full compliance with the ethical standards outlined in the Declaration of Helsinki. All participants signed an informed consent form before the experiment and received monetary compensation after study completion.

**TABLE 1:** Characteristics of the individuals with mild depression and healthy controls.

	Mild depression (*n* = 24)	Healthy controls (*n* = 24)
Age (years)	20.96 ± 1.95	20 ± 2.02
BDI-II score	17.63 ± 3.41	4.63 ± 3.00
**Sex**		
Female	6	9
Male	18	15

*Data are presented as the number or mean ± standard deviation. BDI-II, Beck Depression Inventory test-II.*

### Materials and Procedures

The stimuli used in the experiment were derived from the China Facial Affective Picture System (Gong et al., 2011), a subsystem in the standardized emotional stimuli picture system. We selected pictures of 45 neutral faces and 15 negative faces, including three each of angry, sad, disgusted, surprised, and fearful faces. The experiment consisted of two blocks, emotional block (Emo_block) and neutral block (Neu_block). Each block contained 15 trials. Each trial in the Emo_block contained an emotional expression and a neutral facial expression picture. Each trial in the Neu_block contained two pictures of neutral facial expressions. Each picture appeared randomly on either the right or left side of the screen. All faces were presented without hair, glasses, beards, or other facial accessories, and the two facial expressions used in each trial were combined into one image and presented on the screen. All 30 images were processed with the Adobe Photoshop CS6 software (Adobe Systems Incorporated, San Jose, CA, United States), and the size (1,280 × 738 pixels, 10.84 × 6.25 cm) and gradation were made uniform (Figure 4).

**FIGURE 4:** Representative picture from the Neu_block **(Left)** and Emo_block **(Right)**.

Instructions were displayed on the screen before the beginning of each block. Further, four practice trials identical to the real trials were included to ensure that all participants understood the experimental procedures. Each trial was presented for 6 s. A black background was also presented for 2 s between every two trials. The participants were comfortably seated 60 cm from a 17-inch liquid crystal display monitor with a resolution of 1,024 × 768 and instructed to view each trial freely. A 2-min rest period followed the Neu_block, which was followed by the Emo_block. The whole protocol took approximately 7 min.

### EEG Acquisition and Data Preprocessing

Electroencephalography signals were collected using a 128-channel HydroCel Geodesic Sensor Net (Electrical Geodesics, Inc.). The EEG electrodes were placed according to the HydroCel Geodesic Sensor Net128 Channel Map (Version 1.0) and referenced to Cz. The impedance of all electrodes was maintained below 60 kΩ (Ferree et al., 2001), and EEG signals were continuously recorded at a sampling frequency of 250 Hz. Because the signal gathered between two trials was not valid, each participant’s continuous EEG signals were divided into 30 6-s segments according to marks in the time series. All EEG signals were high-pass filtered at a 0.5-Hz cutoff frequency and low-pass filtered at a 70-Hz cutoff frequency. Eye movement and muscle activity artifacts were discarded using Net Station Waveform Tools. Furthermore, because ocular artifacts are presented in the frequency band between 0 and 16 Hz, they overlap with the alpha rhythm frequency band (8–13 Hz). This study, therefore, used FastICA to eliminate ocular artifacts, as this approach has previously been shown to be effective in delineating between overlapping frequency bands (Hu et al., 2011). We used MATLAB R2010a (Mathworks, Natick, MA) to process all data.

## Results

### Results of Network Analysis

In this section, our results show a significant difference in the small-world property between the two groups by showing the relationship between the small-world property and the thresholds of the two groups (Small-World Property section); statistical analysis of the mean clustering coefficient for each electrode was performed to determine the specific distribution of functional connectivity differences between the two groups in the brain (Statistical analysis of the mean clustering coefficient for each electrode section). In The Topological Structures of the Networks section, we visualized the functional connectivity differences between the two groups using coherence as an example.

#### Small-World Property

Figure 5 shows the mean small-world index S as a function of threshold T for the two groups. For coherence, a significant difference between the two groups was found in the delta band under Neu_block and in the theta band under Emo_block. The value of *S* in the mildly depressed group was significantly lower than that in the healthy control at most of the *T*-values points (indicated by asterisks). For the correlation, PLV, and PLI, we found a similar difference only in the delta band under both blocks.

**FIGURE 5:** The mean small-world index S as a function of the threshold T for the two groups under Neu_block and Emo_block. For the four metrics of coherence, correlation, phase locking value (PLV), and phase lag index (PLI), the values of S in the mildly depressed group were significantly smaller than those in healthy controls. The title of each subgraph is denoted as “metric_band_block.” The horizontal axis presents different thresholds. The values under asterisks (*) denoted the values of *S* at different thresholds when the difference between two groups was significant at these thresholds. **The value of *p* smaller than 0.05; *the value of *p* between 0.05 and 0.1.

In addition, from the separate analysis of γ and λ, we found that the γ of both groups was greater than 1, but the difference between the groups was not significant. The λ of both groups was less than 1 and close to 1, indicating that the brain networks of both groups showed small-world characteristics; however, the λ of the mild depression group was significantly higher than that of the healthy control group, showing that the functional brain network of the mild depression group deviated from the small-world network.

#### Statistical Analysis of the Mean Clustering Coefficient for Each Electrode

Table 2 shows the statistical analysis of the mean clustering coefficient based on independent samples *t*-tests for each electrode for coherence and PLV under Neu_block and Emo_block. For both metrics, we observed a similar pattern, that is, in the delta band, the clustering coefficient of the mild depression group was significantly higher than that of the healthy control group for the electrodes distributed in the temporal and frontal regions, but the results were exactly the opposite for the electrodes distributed in the central and parietal–occipital regions; in the beta band, the mild depression group had significantly lower clustering coefficient in the parietal–occipital region than the healthy controls under Neu_block and Emo_block, and the difference was mainly found in the right hemisphere. We observed a different pattern for correlation. Differences between the two groups were observed in all five bands, and we listed those common electrodes on which there are differences between the two groups in the five bands in Table 3. Similarly, the mild depression group had a significantly lower clustering coefficient than had healthy controls under Neu_block and Emo_block, and the differences were mainly found in the parietal–occipital region of the right hemisphere. The above statistical analysis was performed at a threshold T of 0.15. For the PLI, no differences between the two groups were found on all five bands.

**TABLE 2:** Statistical analysis of clustering coefficient using coherence and PLV (*T* = 0.15).

			Neu_block						Emo_block				
Metric	Band	Electrode	N	D	F	P	region	Electrode	N	D	F	P	region
Coherence	Delta	E31	0.326	0.3026	0.007	0.039	LC	*E2*	*0*.*2719*	*0*.*2851*	*2*.*699*	*0*.*022*	*RF*
		E60	0.3855	0.3646	0.016	0.047	LPO	E7	0.3045	0.2837	0.315	0.02	LC
		E78	0.3777	0.3543	0.014	0.039	RPO	E31	0.3287	0.3026	0.032	0.018	LC
		E79	0.3658	0.3394	0.138	0.033	RC	E60	0.38	0.3585	0.311	0.039	LPO
		E89	0.3859	0.3436	19.833	0.017	RPO	E78	0.3729	0.3503	0.101	0.045	RPO
		E111	0.3392	0.3183	0.525	0.043	RC	E89	0.38	0.341	9.471	0.022	RPO
		*E119*	*0*.*3155*	*0*.*3341*	*0*.*25*	*0*.*043*	*RT*	*E119*	*0*.*3096*	*0*.*3308*	*0*.*07*	*0*.*017*	*RT*
		*E126*	*0*.*2842*	*0*.*2995*	*1*.*457*	*0*.*04*	*RF*	*E126*	*0*.*279*	*0*.*2984*	*0*.*045*	*0*.*013*	*RF*
								*E127*	*0*.*2751*	*0*.*2943*	*1*.*959*	*0*.*012*	*LF*
	Beta	E63	0.3572	0.3238	2.605	0.023	LT	E56	0.3515	0.3177	14.499	0.034	LT
		E67	0.3541	0.3313	1.274	0.03	LPO	E60	0.3569	0.3293	7.942	0.033	LPO
		E68	0.3526	0.3303	1.337	0.032	LPO	E63	0.3588	0.319	10.884	0.017	LT
		E69	0.3575	0.329	0.527	0.035	LPO	E67	0.3577	0.3298	5.523	0.019	LPO
		E71	0.3616	0.3381	2.142	0.046	LPO	E68	0.326	0.3291	5.474	0.023	LPO
		E73	0.3492	0.3185	3.887	0.031	LPO	E69	0.3587	0.3254	4.372	0.028	LPO
		E74	0.3593	0.3319	1.998	0.042	LPO	E71	0.3651	0.336	6.753	0.03	LPO
		E77	0.3543	0.3301	2.533	0.047	RPO	E73	0.3512	0.3148	10.285	0.026	LPO
		E78	0.443	0.3195	3.511	0.038	RPO	E74	0.3619	0.3277	5.502	0.025	LPO
		E84	0.3624	0.3353	1.701	0.044	RPO	E77	0.3575	0.3293	4.993	0.038	RPO
		E85	0.3536	0.3255	1.354	0.027	RPO	E78	0.3471	0.3205	6.769	0.049	RPO
		E89	0.3612	0.3148	0.402	0.006	RPO	E84	0.3635	0.3335	4.796	0.043	RPO
		E91	0.3587	0.3293	1.92	0.036	RPO	E85	0.3552	0.3254	3.586	0.032	RPO
		E98	0.3495	0.3223	7.493	0.044	RC	E86	0.3461	0.3155	6.666	0.033	RC
								E87	0.3275	0.3016	7.723	0.043	RC
								E89	0.3622	0.3093	0.288	0.004	RPO
								E90	0.3622	0.3304	4.187	0.036	RPO
								E91	0.3598	0.3281	3.06	0.036	RPO
								E97	0.3606	0.3266	8.773	0.034	RT
								E98	0.3519	0.3187	10.346	0.027	RC
								E110	0.3393	0.3068	12.954	0.043	RC
PLV	Delta	E1	*0*.*302*	*0*.*3188*	*0*.*235*	*0*.*034*	*RF*	E7	0.3408	0.3149	0.277	0.044	LC
		E2	*0*.*3069*	*0*.*3248*	*0*.*117*	*0*.*025*	*RF*	E60	0.4267	0.4026	0.17	0.037	LPO
		E7	0.3437	0.3193	0.007	0.046	LC	E78	0.4173	0.3903	0.099	0.034	RPO
		*E26*	*0*.*3106*	*0*.*3283*	*2*.*938*	*0*.*028*	*LF*	E79	0.4054	0.3772	0.08	0.037	RC
		E31	0.3734	0.3447	0.464	0.018	LC	E80	0.3682	0.3414	0.781	0.048	RC
		E60	0.4225	0.4007	2.591	0.047	LPO	E85	0.4253	0.4017	0.04	0.038	RPO
		E78	0.416	0.3908	0.546	0.042	RPO	E86	0.4168	0.3908	0.55	0.026	RC
		E89	0.4224	0.3796	9.518	0.022	RPO	E87	0.395	0.3682	0	0.037	RC
		E111	0.3775	0.3555	1.77	0.043	RC	E89	0.427	0.3807	14.249	0.016	RPO
		*E119*	*0*.*352*	*0*.*3779*	0.001	0.017	*RT*						
		*E126*	*0*.*3178*	*0*.*3389*	0.326	0.029	*RF*						
		*E127*	*0*.*3124*	*0*.*333*	0.013	0.195	*LF*						
	Beta	E7	0.2751	0.234	2.879	0.036	LC	E78	0.3583	0.3124	0.582	0.017	RPO
		E23	0.2908	0.2573	0.951	0.043	LF	E79	0.3336	0.2936	1.278	0.031	RC
		E46	0.3411	0.2941	3.461	0.041	LT	E82	0.3742	0.3331	0.008	0.042	RPO
		E60	0.3642	0.3238	2.789	0.045	LPO	E85	0.3675	0.329	0.146	0.046	RPO
		E66	0.3705	0.3344	1.202	0.048	LPO	E89	0.3686	0.3038	1.561	0.012	RPO
		E67	0.3717	0.3335	2.427	0.044	LPO						
		E68	0.3713	0.3323	1.961	0.038	LPO						
		E70	0.3745	0.3379	3.355	0.049	LPO						
		E71	0.381	0.337	1.719	0.019	LPO						
		E74	0.3693	0.3232	1.418	0.023	LPO						
		E76	0.3765	0.3367	1.187	0.031	RPO						
		E77	0.3706	0.3262	2.14	0.022	RPO						
		E78	0.3567	0.3066	3.725	0.016	RPO						
		E79	0.3321	0.2893	3.849	0.037	RC						
		E82	0.3733	0.3189	2.234	0.009	RPO						
		E83	0.3784	0.334	1.224	0.018	RPO						
		E84	0.376	0.3317	1.153	0.03	RPO						
		E85	0.365	0.3128	1.226	0.013	RPO						
		E86	0.3526	0.3048	1.947	0.024	RC						
		E87	0.3243	0.2815	5.833	0.024	RC						
		E88	0.3529	0.303	3.609	0.026	RPO						
		E89	0.371	0.2894	0.101	0.001	RPO						
		E90	0.3708	0.3206	0.907	0.012	RPO						
		E91	0.365	0.321	1.094	0.027	RPO						
		E95	0.3565	0.3096	2.015	0.04	RPO						
		E96	0.3577	0.3104	3.751	0.032	RT						
		E97	0.3551	0.3087	4.479	0.034	RT						
		E98	0.346	0.304	6.075	0.042	RC						
		E105	0.3103	0.2674	7.592	0.045	RC						
		E111	0.316	0.2876	10.572	0.031	RC						

*N, mean clustering coefficient of normal control group; D, mean clustering coefficient of mild depression group; F and p, mean *F-* and *P*-value of independent samples *t*-tests. The electrode distribution of the 128-channel Geodesic Sensor Net is in the Section Appendix. The electrodes are divided into eight regions: the left frontal (LF), right frontal (RF), left temporal (LT), right temporal (RT), left central (LC), right central (RC), left parietal–occipital (LPO), and right parietal–occipital (RPO) regions. The italics indicate that the mean clustering coefficient of mild depression group at this electrode is lower than that of healthy control group.*

**TABLE 3:** Statistical analysis of clustering coefficient using correlation (*T* = 0.15).

Neu_block				Emo_block			
Electrode	*F*	*P*	Region	Electrode	*F*	*P*	Region
E30	2.118	0.042	LC	E60	0.74	0.036	LPO
E36	0.068	0.039	LC	E61	0.843	0.04	LPO
E41	0.187	0.043	LC	E65	1.056	0.034	LPO
E42	0.421	0.041	LC	E66	1.638	0.02	LPO
E46	0.152	0.02	LT	E67	0.879	0.013	LPO
E47	0.024	0.04	LC	E68	0.694	0.012	LPO
E53	0.049	0.029	LC	E69	0.159	0.03	LPO
E60	0.005	0.038	LPO	E70	0.928	0.009	LPO
E61	0.066	0.034	LPO	E71	0.506	0.026	LPO
E64	0.134	0.047	LPO	E73	0.009	0.047	LPO
E65	0.01	0.033	LPO	E74	1.822	0.012	LPO
E66	0.313	0.026	LPO	E76	1.521	0.01	RPO
E67	0.06	0.023	LPO	E77	0.87	0.006	RPO
E68	0.012	0.026	LPO	E78	0.02	0.006	RPO
E69	0.088	0.018	LPO	E79	0.102	0.01	RC
E70	0.044	0.006	LPO	E82	1.055	0.019	RPO
E71	0.463	0.016	LPO	E83	3.964	0.029	RPO
E73	0.64	0.022	LPO	E84	1.443	0.01	RPO
E74	0.012	0.007	LPO	E85	0.561	0.008	RPO
E76	0.212	0.008	RPO	E86	1.404	0.009	RC
E77	0.112	0.005	RPO	E87	0.156	0.046	RC
E78	0	0.007	RPO	E88	1.072	0.043	RPO
E79	0.002	0.016	RC	E89	7.387	0.005	RPO
E82	0.097	0.009	RPO	E90	2.974	0.023	RPO
E83	0.839	0.005	RPO	E91	1.522	0.015	RPO
E84	0.005	0.015	RPO	E92	1.002	0.016	RC
E85	0.135	0.014	RPO	E93	0.404	0.045	RC
E86	0.03	0.023	RC	E94	0.374	0.047	RPO
E87	0.268	0.047	RC	E97	1.489	0.036	RT
E88	0.068	0.028	RPO	E98	0.631	0.042	RC
E89	3.717	0.002	RPO	E104	0.133	0.045	RC
E90	0.048	0.024	RPO	E107	1.632	0.04	RT
E91	0	0.019	RPO				
E92	0.241	0.038	RC				
E93	0.021	0.031	RC				
E94	0.011	0.03	RPO				
E95	0.512	0.028	RPO				
E97	0.027	0.042	RT				
E98	0.022	0.031	RC				
E104	0.115	0.033	RC				
E105	1.097	0.031	RC				
E107	0.019	0.034	RT				
E110	0.694	0.023	RC				

**F* and *p*, mean *F*- and *P*-value of independent samples *t*-tests. The electrodes are divided into eight regions: the left frontal (LF), right frontal (RF), left temporal (LT), right temporal (RT), left central (LC), right central (RC), left parietal–occipital (LPO), and right parietal–occipital (RPO) regions.*

#### The Topological Structures of the Networks

In order to visualize the distribution of coherence differences between the two groups, we plotted the topological structures of functional networks between the mild depression group and healthy controls at a threshold of 0.1 in the delta band under Neu_block. Figure 6 was drawn based on the absolute value obtained by subtracting one coherence matrix from another one. When the absolute value was greater than the threshold of 0.1, there would be a connection in the figure. At a threshold of 0.1, the difference in coherence between the two groups in the delta band can be clearly seen. Most of the connections are distributed in the central, temporal regions and parietal–occipital region of the right hemisphere, and a few connections are distributed in the frontal region.

**FIGURE 6:** The results of the distribution which was the difference of the coherence in the delta band. Red nodes represent 128 electrodes, and the red lines between nodes show the difference in coherence at the threshold of 0.1. The thicker the red line is, the more the threshold is exceeded.

### Classification Results

To evaluate the proposed CNN classification model, 24-fold cross-validation was adopted. In each fold, the functional connectivity matrices from one control and one participant with mild depression were used for testing, while matrices from remaining participants were utilized as training data and for validation. In each fold, the functional connectivity matrices of another mild depression and healthy control participants were used for validation. The functional connectivity matrices of the remaining 44 participants were used for training. This strategy allowed us to avoid records from one participant being divided into both training and test sets and, thus, yielding a falsely high classification accuracy. The classification performance of the validation data was used for selecting the hyperparameters (such as learning rate, learning rate decay, regularization coefficient, number of iterations, weight initialization, etc.) and as a stopping criterion in training to avoid overfitting of the training data.

#### Classification Performance of the Four Functional Connectivity Matrices Using the CNN

We assessed the classification accuracy of the functional connectivity matrices using our CNN method. Since the initial weights of CNN were randomly initialized and different initial weights will train a slightly different model, we repeated the training and testing procedures nine times and calculated the mean and standard deviation of nine test accuracy for further analysis. Coherence performed best under the Neu_block and Emo_block (77.78% for the two blocks). The second highest classification accuracy was achieved with the PLV (74% in the gamma band for the Neu_block, 73.33% in the delta band for the Emo_block). Correlation yielded a 71.46% accuracy for the Neu_block and a 65.83% accuracy for the Emo_block. The PLI achieved the lowest accuracy for both the Neu_block (63.41%) and the Emo_block (55.60%). The classification accuracy of each functional connectivity matrix is shown in Table 4A.

**TABLE 4:** The classification accuracy of each band.

**(A)** The mean accuracy and standard deviation in each functional connectivity matrix using the CNN for the Neu_block and Emo_block.											

		**Accuracy (acc) % and standard deviation (std) %**									
		**Neu_block**					**Emo_block**				
		**Delta**	**Theta**	**Alpha**	**Beta**	**Gamma**	**Delta**	**Theta**	**Alpha**	**Beta**	**Gamma**

Coherence	acc	77.78	75.88	68.64	75.91	75.77	74.48	72.10	72.67	75.57	77.78
	std	1.87	2.17	3.65	1.76	1.86	1.35	4.69	1.86	2.18	2.22
Correlation	acc	70.69	71.33	71.17	70.93	71.46	65.83	60.59	60.94	63.60	63.60
	std	4.30	3.92	3.68	4.19	3.38	3.92	5.51	5.26	5.18	4.94
PLV	acc	71.23	70.93	71.87	66.82	74.00	73.33	71.71	62.64	56.00	64.75
	std	2.12	2.83	3.37	4.50	5.05	1.94	2.88	4.08	3.18	7.11
PLI	acc	61.79	62.27	63.41	61.88	62.16	51.61	50.68	50.73	52.85	55.60
	std	3.89	3.55	3.02	3.33	4.21	2.37	1.10	0.66	1.61	2.82

**(B)** The highest classification accuracy obtained by inputting the feature vector corresponding to each functional connectivity metric into the four classic classifiers (BN, LR, kNN, and RF) in the Neu_block and Emo_block.										

	**Accuracy %**									
	**Neu_block**					**Emo_block**				
	**Delta**	**Theta**	**Alpha**	**Beta**	**Gamma**	**Delta**	**Theta**	**Alpha**	**Beta**	**Gamma**
Coherence	57.22	50	51.67	56.67	61.53	53.47	54.86	51.94	57.78	61.94
Correlation	47.08	49.03	46.81	51.39	52.64	48.19	47.78	47.5	51.39	47.78
PLV	53.19	50	49.03	58.61	60.14	54.31	53.75	49.17	53.06	50.97
PLI	54.72	52.08	52.50	54.03	53.75	56.39	51.67	51.81	53.61	51.25

Receiver operating characteristic (ROC) curves are commonly used to present the results of binary decision problems in machine learning (Davis and Goadrich, 2006). AUC is the area under an ROC curve and has a value between 0 and 1, with a greater AUC value indicating a better classification ability of the model. In order to compare the classification performance of the four input forms more intuitively, ROC curves for four functional connectivity matrices were obtained in the delta, theta, alpha, beta, and gamma bands. These are shown in Figures 7A–E. From these ROC curves, we were able to obtain the same results as those displayed in Table 4A.

**FIGURE 7:** The receiver operating characteristic (ROC) curves of four functional connectivity matrices [coherence (Coh), correlation (Corr), phase locking value (PLV), and phase lag index (PLI)] obtained in the delta **(A)**, theta **(B)**, alpha **(C)**, beta **(D)**, and gamma bands **(E)**, as well as the three-channel input **(F)**. The shaded area in the graph is the result of each measure, and the solid line in the shadow is the average result of nine measures. Neu, neutral picture condition; Emo, emotional picture condition.

#### Performance Comparison Between Our Method and the Self-Established Baseline

In order to further demonstrate the efficiency of our model, we input the four functional connectivity metrics into the four classic classifiers that are widely used in computer aided detection systems for depression (Hosseinifard et al., 2013; Li et al., 2016a; Cai et al., 2018), namely, BayesNet (BN), logistic regression (LR), k-nearest-neighbor (kNN), and random forest (RF), to classify participants into one of two classes, mild depression or healthy. The accuracy obtained from these four classifiers served as the baseline. These classifiers all used the default parameter values implemented in Weka (Witten et al., 1999). The values of *k* used in kNN were 1, 5, and 10. The evaluation method we used herein for classification accuracy also underwent 24-fold cross-validation. Since the inputs for the above four classifiers were feature vectors, we calculated the mean value of all elements in the functional connectivity matrix for each trial, and the mean value for all trials constituted an N × 1 (N represents the number of trials) vector that was then input into the above four classifiers for classification. We only show the highest classification accuracies among the four classifiers in Table 4B.

Table 4B revealed that when functional connectivity metrics were input to the classic classifiers in the form of a feature vector, the recognition rates obtained were obviously lower than the accuracy of the coherence, correlation, and PLV obtained using the CNN. This fully demonstrated the improvements in classification accuracy that our method provided compared to the self-established baseline when the functional connectivity metrics were input into the CNN in the form of 2D data for classification. However, this improvement did not appear in the PLI of the Emo_block.

#### Classification Performance of the Three-Channel Functional Connectivity Matrix

As described above, for each functional connectivity matrix, we used the three bands of the top three classification performance as the R, G, and B channels to generate a three-channel image. We then input this three-channel image into the CNN for it to learn and classify. The bands used for each functional connectivity matrix are shown in Table 5.

**TABLE 5:** The bands used for each functional connectivity matrix in the Neu_block and Emo_block.

	Coherence	Correlation	PLV	PLI
Neu_block	Delta, beta, theta	Gamma, theta, alpha	Gamma, alpha, delta	Alpha, theta, gamma
Emo_block	Gamma, beta, delta	Delta, beta, gamma	Delta, theta, gamma	Gamma, beta, delta

The classification accuracy and ROC curves for the three-channel functional connectivity matrix obtained using the CNN are shown in Table 6A and Figure 7F. Compared with the results of the single channel, the three-channel functional connectivity matrix, which integrated information from three frequency bands, slightly increased the classification accuracy of coherence and correlation in the Neu_block and Emo_block. However, there was no increase in the PLV or PLI accuracy, which performed similarly to a single-channel construct. Figure 8 displayed the comparison of the results of the delta, theta, alpha, beta, and gamma bands, as well as the three-channel coherence that performed the best among the four functional connectivity matrices. The obvious accuracy improvement of coherence through integrating three EEG frequency bands can be observed in Figure 8.

**TABLE 6:** The classification accuracy of the three-channel input form.

**(A)** The mean classification accuracy and standard deviation of the three-channel functional connectivity matrix obtained using the CNN.				

	**Accuracy % ± standard deviation %**			
	**Coherence**	**Correlation**	**PLV**	**PLI**

Neu_block	**78.39** ± 2.62	**71.68** ± 2.51	71.54 ± 4.79	63.12 ± 3.10
Emo_block	**80.74** ± 1.48	**66.93** ± 3.06	65.80 ± 4.57	53.63 ± 2.48

**(B)** The highest classification accuracy obtained by inputting the three-band feature vector corresponding to each functional connectivity metric into the four classic classifiers (BN, LR, kNN, and RF) in the Neu_block and Emo_block.				

	**Accuracy %**			
	**Coherence**	**Correlation**	**PLV**	**PLI**

Neu_block	57.92	51.81	49.72	54.03
Emo_block	54.72	46.81	53.47	51.39

*Bold indicates that the accuracy obtained based on the three-channel functional connectivity matrix is higher than that of single channel in Table 4 (A).*

**FIGURE 8:** Comparison of the accuracy of each band and three-channel image for coherence (Coh).

**FIGURE 9:** The electrode distribution of 128-channel Geodesic Sensor Net.

We also applied the three-channel strategy to the functional connectivity metrics in the form of feature vectors. The functional connectivity metrics on the three bands shown in Table 5 formed an N × 3 feature vector (N represents the number of trials, and three represents the three bands) that was input into the four classic classifiers for classification. The classification accuracies (the highest classification accuracy among the four classifiers) are shown in Table 6B. Compared to the accuracy of the single band that was obtained using the classic classifiers shown in Table 4B, no improvement was provided. This demonstrated that the feature vector form of the functional connectivity metrics did not exhibit the advantages that integrating the three channels in the classic classifiers did and further confirmed the benefits of combining the CNN with functional connectivity matrices.

## Discussion

In the present study, we first illustrated the abnormal organization of functional connectivity network in mild depression by graph theory. Second, we proposed a novel approach of using a CNN to process functional connectivity matrix data in order to identify individuals with mild depression.

### The Differences in the Small-World Network Between the Mildly Depressed Group and the Normal Control Group

Through graph theory, we found that the small-world index of the mild depression group was significantly lower than that of the healthy control group. Small-world networks are characterized by a high clustering coefficient and a short path length (Watts and Strogatz, 1998), while the mild depression group has a lower clustering coefficient and a larger characteristic path length than the healthy control group, indicating that the functional brain networks of the mild depression group deviate from small-world networks. These findings were consistent with previous neuroimaging studies using graph analysis to study depression (Leistedt et al., 2009). The lower clustering coefficient of the mild depression group implies that the local connectedness of networks in mild depression is relatively spared. In addition, short path lengths ensure effective interregional integrity or prompt information transmission in brain networks, which constitutes the basis of cognitive processes. Thus, the increase in the path length associated with the disease may be attributed to the degeneration of fiber bundles for information transmission (Bai et al., 2012).

In addition, the statistical analysis results of the clustering coefficients for each electrode showed that the difference between the two groups was mainly found in the parietal–occipital region of the right hemisphere. The study has shown that the right hemisphere is hyperactive in depression (Hecht, 2010). The parietal region and the right occipitotemporal cortex are the locations of the amygdala and hippocampus. Positron emission tomography studies have shown that the resting blood flow of the amygdala in patients with major depression increased by about 6% (Drevets et al., 1992). Jin et al. (2011) observed an abnormal hyperactive amygdala in depressed adolescents compared to healthy controls. In addition, research reported that the hippocampal volume of depressed patients was significantly reduced compared with healthy controls and the hippocampal neurons of these patients atrophy (Lee et al., 2002). Our findings are consistent with these previous results.

However, it is worth noting that, in the delta band, the clustering coefficient of the mild depression group was higher than that of the healthy control group in the frontal area. Some researchers have suggested that one function of prefrontal cortex is to modulate or inhibit amygdala activity (Davidson, 2004). Ochsner et al. (2002) reported a strong inverse relationship between activation of the prefrontal cortex and the amygdala when subjects were requested to voluntarily downregulate their negative affect. Our results and previous findings suggest abnormal frontal activity in mild depression.

Moreover, through the analysis of small-world properties and clustering coefficients, it is found that the difference between the two groups was mainly in the delta band. Knyazev (2012) reported that delta oscillations are prominent only in early human development stages and during slow-wave sleep. In waking adults, delta oscillations are overshadowed by more advanced processes associated with higher-frequency oscillations. However, delta oscillations are more pronounced in pathological states caused by detrimental environmental factors, developmental pathology, or damage to brain tissue, such as depression.

### Coherence Recognizes Mild Depression Best

In the present study, we used different methods to construct functional connectivity matrices and compared the performance of four of these to identify cases of mild depression. Our results demonstrated that coherence was most effective in identifying mild depression using a CNN.

By using Eqs. (1) and (3), we determined that the PLV was the amplitude-normalized coherence. There are two perspectives on coherence and PLV. Researchers who support the use of the PLV often claim that the phase synchronization reflected by the PLV is more stringent than that for coherence because the latter confuses the consistency of the phase difference with amplitude correlation. This may be true from a mathematical point of view, but one might argue that when there are no amplitude correlations, it would be more “difficult” to get a meaningful non-zero coherence value in the absence of consistent phase differences. For example, when none of the separately observed cross-spectral density estimates has phase synchrony, even if there is perfect amplitude correlation, the expected value of the vector averages will be relatively small. On the other hand, if cross-spectral densities of all individuals are estimated to be strongly phase-synchronized, the expected value of their vector averages is still perceptible even in the absence of amplitude correlations. In addition, those in support of using the coherence also believe that in the case of coherence, the observations with large-amplitude products are given stronger weight, meaning they are favoring those observations that have a higher-quality phase difference estimate. This actually assumes that a higher amplitude reflects a higher signal-to-noise ratio of the source of interest, and thus a better-quality phase estimate (Bastos and Schoffelen, 2016). A better-quality phase estimate may result in coherence achieving better classification performance than the PLV when using a CNN. However, the classification performance of the PLI in our CNN was relatively poor. This may be because the PLI is sensitive to the chosen length of the selected epochs (Fraschini et al., 2016), which was 6 s in the present study. This may have been too short to allow the PLI to stabilize.

### The Three-Channel Functional Connectivity Matrix Improved Recognition Performance

Based on the data shown in Tables 4A, 6A, it is clear that the three-channel functional connectivity matrix used herein improved the accuracy of coherence and correlation slightly, achieving an accuracy similar to that of single channels for the PLV and PLI. We suspect that human cognitive processes involve different EEG rhythms, making it reasonable that neural networks learn the information contained across several integrated EEG spectrums. However, this conjecture requires further, future verification using additional data sets.

## Conclusion and Future Work

In summary, the present study first illustrated that some abnormal organizations in the functional connectivity network of patients with depression also appeared in individuals with mild depression. Specifically, compared with healthy controls, the mild depression group has a larger characteristic path length and a lower clustering coefficient, indicating that the brain functional network of mild depression deviated from the small-world network. Second, we proposed a computer-aided method by which a CNN was used to learn information relevant to the functional connectivity matrices evident in individuals with mild depression such that they could be readily identified. This is an innovative approach other than the existing graph theory for the use of functional connectivity matrices for depression recognition. We primarily considered functional connectivity matrices that reflect altered brain functional connectivity in patients with mental illnesses using a 2D data structure given the advantages of CNNs in processing 2D datasets. The classification results of our method showed that coherence, correlation, and the PLV can effectively recognize mild depression using a CNN and that the recognition performance of coherence was superior to the other functional connectivity metrics, obtaining a classification accuracy of 80.74%. The proposed method can provide an auxiliary diagnosis of mild depression and offers great promise. In the future, we are committed to implement this method as an online depression detection system. Once an individual’s EEG signal is collected, it is used to determine whether the individual has mild depression, a disease that is not easily detectable and diagnosable. This approach may be used to improve and hasten the detection of individuals with mild depression, ultimately permitting quicker treatment.

While the present study offers significant benefits, it has some limitations that warrant discussion. First, in addition to the functional connectivity matrices used in the present study, there are other various connectivity metrics available, such as the imaginary part of coherency (Nolte et al., 2004), partial directed coherence (Baccalá and Sameshima, 2001), directed transfer function (Kamiñski et al., 2001), phase slope index (Nolte et al., 2008), and Geweke’s extension of Granger causality to the frequency domain (Brovelli et al., 2004). Further investigation of these metrics and their ability to detect the signatures of mental illnesses such as depression must continue in the future. Second, we used the functional connectivity metrics generated by all 128 pairs of electrodes available to us here. It is necessary to further explore which electrodes most obviously dictate functional connectivity matrix differences between healthy control individuals and those with mild depression. This would allow greater reductions to the number of electrodes used for classification and pave the way for real-time, online depression detection.

## Data Availability Statement

The datasets generated for this study are available on request to the corresponding author.

## Ethics Statement

The studies involving human participants were reviewed and approved by the Ethics Committee of Lanzhou University Second Hospital. The patients/participants provided their written informed consent to participate in this study.

## Author Contributions

XL and RL conceived the project idea. BH supervised the project. XZ provided critical suggestions for the statistical analysis. RL and YW performed the experiments and surveyed the literature, to check whether our findings were consistent with previous publications, and wrote the manuscript.

## Conflict of Interest

The authors declare that the research was conducted in the absence of any commercial or financial relationships that could be construed as a potential conflict of interest.

## Footnotes

1 https://www.who.int/mental_health/management/depression/en/

2 http://www.nbtwiki.net/

3 https://github.com/Lasagne/Lasagne

## Appendix

The electrode distribution of 128-channel Geodesic Sensor Net (Figure 9).
Left frontal region (LF, number = 13): E32, E26, E23, E19, E12, E25, E22, E18, E21, E27, E24, E127, E128;
Right frontal region (RF, number = 13): E1, E2, E3, E4, E5, E8, E9, E10, E14, E123, E124, E126, E125;
Left temporal region (LT, number = 17): E33, E34, E38, E39, E40, E43, E44, E45, E46, E48, E49, E50, E51, E56, E57, E58, E63;
Right temporal region (RT, number = 17): E122, E116, E121, E115, E109, E120, E114, E108, E102, E119, E113, E101, E97, E107, E00, E96, E99;
Left central region (LC, number = 16): E7, E13, E20, E28, E29, E30, E31, E35, E36, E37, E41, E42, E47, E52, E53, E54;
Right central region (RC, number = 16): E106, E112, E118, E117, E111, E105, E80, E110, E104, E87, E103, E93, E98, E92, E86, E79;
Left parietal–occipital region (LPO, number = 13): E59, E60, E61, E64, E65, E66, E67, E68, E69, E70, E71, E73, E74;
Right parietal–occipital region (RPO, number = 13): E91, E85, E78, E95, E90, E84, E77, E94, E89, E83, E76, E88, E82.
